The article "Analysis and Improvement of Nursing Quality Based on Standardized Information Integration" was retracted in 2023. Reasons: signs of a paper mill; suspected computer-generated content; unreliable results or conclusions; concerns about the data.

# Analysis and Improvement of Nursing Quality Based on Standardized Information Integration

**DOI:** 10.1155/2022/9172416

**Published:** 2022-02-11

**Authors:** Huixia He, Huiling Li, Kong Qiao, Bin Hao, Dong Yu

**Affiliations:** ^1^Hand and Foot Microsurgery, Bayan Nur Hospital, Bayannur, Inner Mongolia 015000, China; ^2^Department of Mathematics and Computer, Hetao College, Bayannur, Inner Mongolia 015000, China; ^3^Department of Information Engineering, Bayan Nur Hospital, Bayannur, Inner Mongolia 015000, China

## Abstract

Information is becoming increasingly important in social development, and the medical industry's informatization has made significant progress. This paper evaluates the role of nursing informatization in improving nursing quality management by analyzing and comparing changes in nursing quality before and after the implementation of nursing informatization. Using modern computer network technology to evaluate nursing quality, monitor the implementation of nursing management plans, and control nursing quality links in real time has helped to promote and improve nursing quality. The integration mode of the existing hospital information system is sorted out and standardized according to the requirements of refined hospital management. We can optimize the overall architecture of the hospital information system, reduce the tight coupling between business systems, support rapid integration and flexible expansion of business systems, and lay a foundation for the cooperation and data sharing of medical resources in and out of the hospital by establishing a hospital information platform based on standardized specifications.

## 1. Introduction

With the rapid development of science and technology, the introduction of computers into the medical industry has become the basis of modern hospital management. For hospitals, medical quality is not only the lifeline, but also the main core of nursing management. Nursing quality is directly related to the medical level of hospitals [1]. The establishment of electronic information system in hospital is an indispensable tool and means in hospital management and an important measure to achieve the goal of modern hospital management [2]. Traditional nursing management is prone to the problems of slow information turnover, untimely business supervision, and poor standardization of organization and management. With the continuous improvement of information system, the rational use of informatization makes it a powerful helper for nursing managers [3]. The members of the quality control organization are composed of hospital leaders, the nursing staff are not involved, and the quality control members do not understand the work status of grass-roots nursing staff [4]. Therefore, the quality control organization cannot fully consider some problems. From the perspective of nursing staff, the inspection team is a burden [5]. Therefore, in the face of examination, it is only regarded as a form. On the surface, the quality of nursing is high. However, in fact, there are all kinds of problems in nursing work. With the deepening of the reform of public hospitals, the original information infrastructure and business systems of many hospitals have been unable to meet the business needs of hospital fine management, especially in information integration and data analysis and utilization. Nursing quality is one of the important contents in hospital management, and the nursing quality management system includes quality construction, quality supervision, monitoring, evaluation, and quality continuous improvement [6].

Nursing is an important part of hospital work, and clinical nursing information systems have become one of the components of hospital information systems, and their development has a direct impact on hospital and community health service management and effectiveness [7]. At this time, hospital development is heavily focused on information technology. Information collection, preservation, transmission, analysis, and processing are all aided by hospital informatization's progress toward electronization, mobility, and barcodes. It is convenient and efficient, increases accuracy and effectiveness, and reduces errors [8]. Because of its ease of data acquisition, the mobile nursing system is a new research direction in information integration and sharing application. In the regional context, a hospital information platform is a critical link in the realization of patient-centered interinstitutional medical information sharing and business collaboration services [9]. The core of nursing management is improving nursing quality and meeting patients' growing health needs. Creating and relying on an information platform is an effective way to promote continuous medical quality improvement.

The traditional business process-driven software development model and point-to-point business system integration model have been unable to meet the new requirements of hospital data planning, and a new model needs to be found for medical information construction [10, 11]. At present, Chinese hospitals are vigorously developing informatization construction so that informatization can better serve patients. Therefore, in the informatization construction, a series of models, application strategies, and methods have been formed [12]. “Hospital information platform based on electronic medical records” refers to the medical information sharing and business cooperation platform connecting clinical information system and management information system based on information collection, storage, and centralized management of patient electronic medical records [13]. It is the basis and carrier of unified integration, resource integration, and efficient operation among different business systems in the hospital. The hospital information platform based on electronic medical records has become an important support to overcome the obstacles of hospital information construction [14]. Hospital informatization construction is gradually shifting from business process software system as the core to a brand-new architecture model based on data planning and information platform as the core [15]. On the basis of perfecting the quality management system and establishing the quality control organization, this paper develops and applies nursing management assistant decision-making, head nurse electronic workbook, nursing electronic medical record, and nursing mobile ward round software step by step by using modern computer network technology. In this paper, a nursing quality basic data collection, management plan implementation, quality analysis and monitoring, and risk prospective prevention system was established, and the continuous improvement of nursing quality was realized.

## 2. Related Work

Literature [16] believes that the biggest problem facing the application of mobile nursing system technology is that there are greater difficulties in the seamless integration of clinical information and real-time interconnection, which requires continuous optimization and improvement. Literature [17] shows that most tertiary hospitals in China have built a hospital information management system, and its development and application are developing in depth, from focusing on financial operation management, gradually extending to clinical applications and management decision-making applications. Literature [18] proposes that the construction of an information system in a hospital can improve efficiency, save resources, improve service quality, and increase benefits, which is an important way to become a modern hospital. Literature [19] pointed out that many hospitals have implemented inpatient nurse workstations, but they only deal with simple tasks such as doctor's order transfer, printing, and expense entry. Literature [20] developed a nurse human resource planning system based on a microcomputer. Literature [21] pointed out that the coverage of the front-end sensors of the hospital information system and the popularity of networking have become a prerequisite for its development. Therefore, at the level of information collection, it must be three-dimensional, full range, full coverage, and try to avoid omissions and leave no dead ends. Literature [22] believes that in order to realize medical informatization, it is necessary to realize that the human, financial, and material information of medical institutions, the electronic medical records of patients, the results of various testing and inspection equipment, and other complicated data information can be eliminated in this hospital information system. *Obstacle to Flow*. Literature [23] tries to design, develop, and demonstrate the planning, investment and control system of auxiliary hospital management. Literature [24] believes that the hospital information system is a kind of enterprise management system, but different from the general enterprise management system, it serves doctors and patients. Literature [25] pointed out that informatization construction is an important part of medical reform, and hospital informatization construction is imperative. In order to realize all-round medical informatization, medical data standardization must be at the forefront. Literature [26] mentioned that due to the change of medical model and the implementation of holistic nursing, the patient's demand for nursing is increasing, which makes the situation of insufficient nursing human resource allocation even more serious. Literature [27] believes that the developers of modern clinical information systems did not focus on the nursing profession in isolation, but instead focused on the establishment of a multidisciplinary system aimed at supporting a wide range of information systems. An information system with extensive patient clinical data can provide support for quality assessment and improvement of nursing and clinical treatment. Improving the quality of care and meeting the growing health needs of patients is the core of nursing management. Establishing and relying on an information platform is an effective way to promote continuous improvement of medical quality. Therefore, it is of great significance to establish a nursing information system. The information database of comprehensive nursing information platform constructed in this paper has strong expansibility and advanced technology. Through the application of information technology, the nursing quality management can be guaranteed so as to maximize the safety of patients, improve the present quality of patients, and improve the management level of nursing managers. Save nurses' indirect nursing time and improve the standardization of nursing records. Electronic nursing record sheet is superior to handwritten record sheet in standardization, timeliness, and accuracy. The nursing information system improves the level of nursing quality management.

## 3. Methodology

### 3.1. Nursing Information System

The comprehensive information platform for nursing is a dynamic and visual comprehensive information platform for nursing management, which is supported by the hospital information system and focuses on daily management objectives such as doctor's advice management, electronic nursing medical records, and nursing quality management [28]. The nursing information system consists of four software. The overall design is based on the relatively independent and interrelated functions of four software, collecting basic data of nursing quality on the basis of nursing management decision-making software and nursing electronic medical record software, supervising the implementation of nursing management plan by means of head nurse electronic workbook software, automatically monitoring the nursing process of patients by using nursing mobile rounds software, and promoting the continuous improvement of nursing quality by computer. The nursing information system is shown in Figure 1.

Traditional nursing management has some flaws, such as poor organizational and management standardization, slow information turnover, and so on. Currently, the information system is improving all the time, and nursing managers can improve management quality by using information management in a scientific and rational manner. Nurses and computers make up a nursing information system, which collects, stores, and processes nursing management and business technical data [29]. In the development of hospitals, information technology is the most important factor to consider. Informatization in hospitals has progressed to the point where barcodes and electronization are used, making it easier to share and process information. Its benefits include increased efficiency and speed, which not only improves nursing quality but also reduces nursing errors.

The head nurse manages the work manual system and establishes the standard data query field database, and the head nurses and nursing department managers of each department can use it by multiple users with different permissions, and the head nurses can input and query the related nursing management contents of the department. The nursing department can inquire about the contents of all subjects in the whole hospital, but has no right to modify them. The head nurse's handbook is a memorandum of the head nurse's work. The main contents are as follows: (1) Formulating annual, monthly, and weekly nursing work plans and recording annual work summary. (2) Monthly record of self-examination and self-correction of nursing quality. (3) Report nursing defects and corrective measures. (4) Continuous quality improvement plan and measures management. (5) Formulation of risk management projects, implementation of measures and effect evaluation. The function of the system in promoting the continuous improvement of nursing quality is to draft improvement plans according to the nursing quality feedback from the nursing department and the self-discovered undergraduate nursing quality problems and nursing defects, consciously implement improvement measures and self-evaluate the improvement effect.

The electronic nursing medical record system is applied to all nursing staff on the basis of strict authority and safety control. It is mainly used for computer management of nursing documents and real-time monitoring of the whole process of prereminding, in-process supervision, and postevaluation of the writing time limit and writing quality of nursing electronic medical records. Main functions of the system: (1) Management of nursing admission evaluation form, nursing records, temperature list, and so on. (2) According to the time limit of all kinds of records in the nursing medical record writing specification, the computer automatically checks the timeliness and completeness of all kinds of records and reminds nurses in advance. (3) The nursing department queries the nursing medical records of the whole hospital in real time and grasps the nursing quality. And check the timeliness, accuracy, integrity, and other information of nursing medical records automatically counted by computer.

*Mobile Nursing Ward Round System*. On the basis of wireless network coverage in wards, barcode identification of patients' identities, medicines, and test specimens, automatic identification of nursing operation handheld computers is adopted to actively meet the standard requirements of three checks and seven pairs of nursing. It is applied to all nurses, mainly used for drug treatment, patient identity check during specimen collection, and basic nursing operation records. The main functions of the system are as follows: (1) Check the doctor's orders. (2) Check the collection information of test specimens. (3) Vital signs entry. (4) Nursing operation records.

The management assistant decision-making system is applied to the nursing quality control department, which mainly collects the registration, statistics and analysis of the data of previous department nursing quality inspection, nurses' personal business, and theoretical assessment. All data and contents are input after inspection and examination by the nursing department, and the computer automatically summarizes and calculates according to the required query items, and the analysis interface is illustrated with pictures and texts. The head nurse can check the current and historical quality through the network, but has no right to modify it. The main functions of the system are as follows: (1) The entry and statistics of the scores of previous nursing quality examinations in departments. (2) Entry and ranking of personal business and theoretical assessment results. (3) Longitudinal comparison of nursing quality in different periods. (4) Horizontal comparison of nursing quality in different departments. (5) Monthly dynamic analysis of nursing quality. (6) Quality analysis of nursing medical records. (7) Analysis of nursing defects. With the application of nursing management assistant decision-making software, the head nurses can understand the nursing quality problems existing in departments, check the dynamic nursing quality, and compare horizontally by departments or vertically by time, which not only introduces the competition mechanism among the head nurses, but also helps the head nurses to make targeted and timely improvement, which can effectively promote the improvement of nursing quality in the whole hospital year by year.

### 3.2. The Role of Nursing Information System in Promoting Continuous Improvement of Nursing Quality

The greatest advantage of information system is preventive quality improvement, and the focus of continuous quality improvement should be to prevent the occurrence of problems. Only prior quality control can achieve permanent and fundamental quality improvement [30]. At each stage of plan implementation, it is better to focus on preventing defects than to supervise problems.

Change nurses' perceptions of quality management by teaching them that the most important aspect of nursing care is to meet patients' needs as much as possible, rather than forcing patients to adapt to hospital management. Patients should be treated as nursing centers, and all nursing decisions should be made with their input. Reduce conflicts and disputes between doctors and patients by increasing nurses' acceptance of nursing quality control. Nurses can only improve their clinical work execution if they truly understand the assistance and guidance provided by nursing quality control. As a manager, communicate effectively with nurses to gain a better understanding of the practical difficulties and weaknesses that nurses face in their jobs and to address them appropriately in order to improve nurses' satisfaction with nursing quality control. Nurses should abandon the passive nursing mode of the past and actively implement nursing, not just strengthening the aseptic operation of nurses.

Informatization is an effective method for continuous quality improvement. With the help of hospital information system, the information of medical process can be directly collected and processed, the quality situation can be tracked, the quality problems can be found, the quality control can be implemented, and the quality can be evaluated. It is an effective method for continuous quality improvement to transform the traditional quality control after feedback of final quality evaluation into real-time tracking quality control of process quality control.

The scheme design is mainly divided into four parts, namely, input image preprocessing, classification feature selection, classifier training, and character recognition extraction. Its topology is shown in Figure 2.

Through the management of nursing information system, in different stages of nursing quality management, such as planning, implementation, inspection, and processing, the standard data collected by different information systems play their respective functions cooperatively and jointly promote the improvement of nursing quality. After each form, there are quality standards and scores. Inspectors only need to click against the standard, deduct points directly if they fail to meet the standard, and display the unqualified contents in the summary table below, and then the inspectors will write out the problem description and put forward rectification suggestions.

The focus of continuous nursing quality improvement should be on preventing problems rather than checking and correcting them after they occur. The only way to achieve permanent and fundamental quality improvement is to conduct quality control in advance, and the greatest benefit of a nursing information system is preventive quality improvement. Strengthen link control in the implementation process, and ensure timely information feedback to quickly correct errors and avoid negative consequences. Improve quality even more by using a combination of proactive reminders, on-the-job supervision, and postprocess evaluation. Use technological means to improve nursing quality by reforming workflow and preventing errors. A nursing information system can serve as a foundation for quality-improvement decision-making in the long run. Facts and data must be used to make decisions, and improvement measures must be based on facts and data to ensure continuous quality improvement. The nursing quality inspection information is gathered by the management assistant decision-making system. We can quickly identify quality issues, assess the work effect, and determine whether there are opportunities to improve the work and solve problems using the directional analysis of the nursing information system.

Based on the hospital information system, all information data of various departments and nursing processes in the hospital were directly collected and processed. Through the information system, it provides the functions of optimal combination, intelligent judgment and assistant decision-making, tracking quality situation, finding quality problems, implementing quality control, and evaluating quality at any time. It is the development trend of medical quality management in the future and an effective method of continuous quality improvement to transform the traditional quality control after feedback of final quality evaluation into real-time tracking quality control of process quality control. Nursing information system can help nurses use modern tools and means to directly serve patients and improve work efficiency.

### 3.3. Analysis and Improvement of Nursing Quality

First, build a font library for all characters in each font to form a precorrelation template; then normalize the input image data to be recognized according to the resolution of the font library, perform two-dimensional cross-correlation matching between the input data and the prebuilt font library, and take the characters with the maximum correlation in the font library as recognition results for output. Provide business logic methods to the presentation layer. The method itself judges whether the input data is legal and valid and calls the interface of data access layer after verification to realize data addition, deletion, and modification. After execution, return the processing result and processed data to the caller.

The set threshold a is the projection pixel accumulation threshold, and the set threshold *b* is the continuous fracture threshold. Scan the projection result from left to right. When a point less than a value appears in the statistical value of the projection result, it is judged that the point is broken. When the cumulative number of points less than the value of *a* in the projection result is greater than *b*, it is judged that the characters here can be divided.

The bilinear interpolation method only needs the pixel values of 4 adjacent points near the point to be interpolated to be calculated. The calculation process is as follows: Suppose the point to be interpolated is *f*(*u*, *v*), where (*u*, *v*) is the decimal coordinate value; then the 4 adjacent points are *f*([*u*], [*v*]), *f*([*u*] + 1, [*v*]), *f*([*u*], [*v*] + 1), and *f*([*u*] + 1, [*v*] + 1); let *a* = *u* − [*u*], *b* = *v* − [*v*]. The result of one-dimensional linear interpolation in the abscissa direction is

(1) $$\begin{array}{c} \left\{\begin{array}{c} t_{1}=af\left(\left[u\right]+1,\left[v\right]\right)+\left(1-a\right)f\left(\left[u\right],\left[v\right]\right),\\ t_{2}=af\left(\left[u\right]+1,\left[v\right]+1\right)+\left(1-a\right)f\left(\left[u\right],\left[v\right]+1\right). \end{array}\right. \end{array}$$

In the same way, substituting the interpolation result into the ordinate direction for the second one-dimensional linear interpolation, then

(2) $$\begin{array}{c} g\left(x,y\right)=f\left(u,v\right)\\ =bt_{2}+\left(1-b\right)t_{1}. \end{array}$$

A one-dimensional difference template is used for gradient calculation for all pixels in each unit. Suppose the pixel value of each point in the image is *f*(*x*, *y*); then the one-dimensional gradient calculation formula corresponding to each point is as follows:

(3) $$\begin{array}{c} \left\{\begin{array}{c} \Delta_{x}\left(x,y\right)=f\left(x+1,y\right)-f\left(x-1,y\right),\\ \Delta_{y}\left(x,y\right)=f\left(x,y+1\right)-f\left(x,y-1\right), \end{array}\right. \end{array}$$

where Δ_*x*_(*x*, *y*) is the horizontal gradient value, and Δ_*y*_(*x*, *y*) is the vertical gradient value. From the above formula, the one-dimensional difference template matrices used in gradient calculation are [−1 0 1] and [−1 0 1]^*T*^, and the two templates are used to perform convolution calculations on the image data to obtain the one-dimensional gradient information *D*_(*x*, *y*)_(Δ_*x*_, Δ_*y*_) of each point.

From the one-dimensional gradient information of each point, the gradient amplitude *A* (*x*, *y*) and the gradient direction *θ* (*x*, *y*) corresponding to the pixel can be obtained as follows:

(4) $$\begin{array}{c} \left\{\begin{array}{c} A\left(x,y\right)=\sqrt{\Delta_{x}{\left(x,y\right)}^{2}+\Delta_{y}{\left(x,y\right)}^{2},}\\ \theta \left(x,y\right)=\arctan\frac{\Delta_{x}\left(x,y\right)}{\Delta_{y}\left(x,y\right)}. \end{array}\right. \end{array}$$

Data integrity, in general, ensures the integrity of entities, references, and user-defined data, whereas entity integrity and reference integrity are the integrity requirements that databases must meet during the design process. The data usage specification that should be followed in database operations is known as user-defined integrity.

Solving the optimal classification hyperplane of support vector machine is mainly to solve the support vector samples in the sample space. When the sample set satisfies the condition of linear separability, the classification hyperplane equation satisfies the following conditions:

(5) $$\begin{array}{c} y_{i}=\omega x_{i}+b\\ =0. \end{array}$$

Among them, *x*_*i*_ represents the *i*th data point, *y*_*i*_ represents the classification result corresponding to the *i*th data point, *ω* represents the normal vector of the hyperplane, and *b* represents the intercept of the hyperplane to the feature space. According to the logistic regression model, let *y*_*i*_=−1 and *y*_*i*_=1 represent two different classification results.

The hospital information integration platform enables real-time and data consistency between mobile application-specific data centers and clinical data centers. The nursing department or the department's head nurse set and distributed the quality control contents, and the nursing staff listed the quality control contents and presented the existing problems. The quality control personnel went to the department site for quality control and timely entry after receiving the quality control task, which was a problem. Each department's head nurses complete the problem cause analysis and corrective measures, while the nursing department examines quality control issues and improvement effects, as well as tracks and supervises the major issues. After passing this quality control, there will still be an unqualified nursing department to assist in locating the source of the problem, as well as to monitor and supervise shift work until the quality control is passed.

Adopt a layered architecture. Call the services provided by the lower layer, and each layer is built on a more general layer. The advantage of the hierarchical structure of is that the attention is dispersed so that developers can only pay attention to one layer in the whole structure. Decentralized coupling makes it easy to replace the implementation of the original level with a new one, which can reduce the dependence between layers. Logic reuse can be beneficial to the reuse of each layer of logic.

Assuming that the projection point from the sample *x* to the classification hyperplane is *x*_0_, the distance *γ* from the sample to the hyperplane satisfies the following formula:

(6) $$\begin{array}{c} x=x_{0}+\frac{\gamma \omega }{\left\|\omega \right\|}. \end{array}$$

From the above formula, it can be derived that the maximum separation of the classification hyperplane corresponding to the support vector sample is 1/‖*ω*‖; that is, when ‖*ω*‖ is the smallest, the classification distance is the largest to meet the requirements of the optimal classification result of the support vector machine. Taking the classification hyperplane equation as the constraint condition, when the convex quadratic programming problem *f*_*x*_=0.5‖*ω*‖^2^ is satisfied, the required solution can be obtained.

For hospital nursing quality management, the networked nursing quality management system provides an effective platform. Management switched from terminal to link quality control, which improved nursing quality and decreased nursing risk significantly. Simultaneously, disparate and static data will become comprehensive and dynamic, allowing for tracking management to be carried out quickly, accurately, and consistently. To design and develop a comprehensive nursing management information platform, this chapter primarily uses wireless network technology and software development technology. Data connection and data conversion issues between the comprehensive nursing management information platform and other systems are addressed using database association technology. Database association technology can also perform statistical analyses on the system's various data. Also, set up a system for assessing nursing quality. It establishes a reporting system for nursing adverse events and provides a monitoring platform for nursing quality management. It optimizes the nursing management process and improves nursing management quality in the areas of clinical nursing quality index management, forward-looking risk assessment, and nursing management quality.

## 4. Results Analysis and Discussion

Comprehensive nursing information platform highlights nursing modernization and humanized management means. It is beneficial to increase the nursing time of nurses and improve the nursing quality. However, in the past, the simple nurse station could not effectively realize the closed loop of nursing process. Therefore, in the new system, new technologies and methods are added. It can greatly improve the potential safety hazard and improve the phase ratio. The efficiency and quality of nursing management have been improved. The application of hospital informatization has optimized the process and quality of nursing management. Especially, the process and reengineering of key links such as patient identification, doctor's advice handling, and doctor's advice checking can shorten the nursing quality control time, reduce the occurrence of nursing adverse events, and improve the efficiency of nursing management.

The collected effective data were processed by software, and descriptive statistics were made on general data, nursing practice status of patients after general anesthesia, and nurses' mastery of nursing knowledge of patients after general anesthesia by frequency, composition ratio mean, and standard deviation. Sample loss is shown in Figure 3.

The “dictionary database” of various nursing quality standards in the system is summarized and integrated according to a certain logical hierarchy to form a collection of information items with nursing management characteristics. A highly organized and integrated decision support system is formed by using the management information system, which can provide managers at all levels with the required information in an extremely complicated and rapidly changing external environment. Moreover, the system design is open, and the management model design is reasonable, and various statistical information can be quickly obtained, and then Excel tables can be exported for further statistical analysis.

Under the same scale of ensemble, the effect of selective ensemble is better than that of unselected ensemble, which shows that some base classifiers are redundant and the algorithm in this paper is effective. With the increase of integration scale, the improvement of integration effect is not obvious. The possible reason is that the difference caused by the added member classifiers to the whole integrated classifier is getting smaller and smaller. Therefore, when constructing the base classifier, we should comprehensively consider the storage and time overhead allowed in practical application to select the appropriate integration scale. The experimental results are shown in Figure 4.

Taking 4 adjacent segmentation units to form a feature block, the feature vector of 4 × 8 = 32 dimensions can be obtained simultaneously. The normalized resolution of the input character image is 16 × 18, the characteristic block width is 4 × 2 = 8, and the length is 6 × 2 = 12. Taking the scanning step size as 2 pixels, the horizontal direction includes (16 − 8)/2 = 4 block scanning windows, and the vertical direction includes (18 − 12)/2 = 3 block scanning windows. Each scanning window contains 36 feature vectors, a total of 4 × 3 × 32 = 384 feature vectors. The model in this paper and the traditional model were used to carry out statistical experiments on the complications of patients after general anesthesia, and the statistical error rate and the time required for the statistics were compared. The comparison results are shown in Figures 5 and 6.

The superiority of nursing informatization implementation can be proven more accurately and concretely by comparing various special inspection data record indicators before and after the implementation of hospital nursing informatization, and the standardized nursing quality management model provides the foundation. The Clinical Data Repository (CDR) is the foundation of any hospital information system. To achieve rapid storage, retrieval, and reading of clinical data, the patient-centered reconstructed data repository standardizes and optimizes clinical data with different structures and terms. The goal and core of the mobile nursing system's development is to figure out the best way to process clinical data so that data and information can be shared across different clinical manifestations, nursing documents can be generated automatically in real time, and medical staff can record less information.

The concept of nonpunishment management encourages nurses to actively report and eliminate all kinds of worries in the development and application of electronic information for reporting adverse nursing events. At the same time, the system has established permissions for each department's operation. Departments can only see the data and information that their own departments have reported, and the nursing department can only see the data and information that each department in the hospital has reported. When analyzing, discussing, and commenting on adverse events, the nursing management committee follows the principle of confidentiality and does not reveal department information. Common problems will be discussed throughout the hospital, and solutions and measures will be proposed.

The fast and effective electronic statistics function standardizes the text format, which not only improves the efficiency, but also reduces the cost. There are 213 files in 20 folders in nursing management, which reduces the printing of about 1,300 manuals and the file transmission between nursing department and all nursing units for about 180 times throughout the year. The input and analysis of quality inspection data saved 7 working days per month on average. An initial node needs to be randomly selected, and the accuracy of generating the final model is different with different initial nodes. The model generated by traditional genetic algorithm is compared with the model generated by random initialization method. The experimental results are shown in Figure 7.

The construction of hospital information platform should take the opportunity of the maturity evaluation of standardization of hospital informatization interconnection and lay a solid foundation for information exchange, business collaboration, and management decision support inside and outside the hospital. Through standardized information integration, the analysis method of nursing quality can be improved, which is conducive to the improvement of analysis efficiency. The linear regression curve is calculated according to the stepwise multiple linear regression equation, as shown in Figure 8.

The development direction of nursing information system is nursing expert system, hospital nursing integrated management information system, and remote nursing. The tide of mobile medical care is overwhelming, and it has brought huge business opportunities and challenges to wireless, network, storage, security, software, integration, and other fields. This paper developed and utilized nursing information systems such as nursing management decision-making, head nurse's electronic manual, nursing electronic medical records, mobile nursing rounds software, and so on. According to the core system of nursing work, nursing quality indicators, nursing quality management standards, nursing quality standards, nursing quality control methods, and management measures, standardized management concept is transformed into an intelligent nursing quality control system and implemented. According to the research, the number of reported cases of nursing leak blocking incidents decreased. Improve nurses' satisfaction with nursing quality control and patients' satisfaction with nursing service. Nurses' satisfaction with nursing quality control has been significantly improved. Patients' satisfaction with nursing service after informatization is higher than before. The frequency of problems in electronic nursing records is less than that in handwritten records. The nursing information system established in this paper has strong expandability and advanced technology and improves the nursing quality management level.

## 5. Conclusions

This paper can find quality problems in a timely manner, evaluate the work effect, and then analyze whether there is an opportunity to improve the work and solve the problems, and finally promote the continuous improvement of nursing quality through directional analysis of information systems. Nursing management, as an important part of hospital nursing ability, should be grasped at the pinnacle of modern nursing quality in order to discover the characteristics and laws of nursing management. Nursing management can only be implemented if the characteristics and laws are understood. The construction of a standardization system is a time-consuming and systematic process. Clinical nursing quality evaluation indexes are used to reflect the basis, process, and outcomes of nursing quality in a scientific and dynamic way. Scientific evaluation of nursing quality, continuous evaluation and monitoring of nursing quality, continuous improvement of nursing quality, and standardization, specialization, standardization, and refinement of nursing quality management are all carried out based on data. The information database of the comprehensive nursing information platform built in this paper is highly expandable and technologically advanced. At the same time, this paper has completed the design of various functions of the comprehensive nursing management information platform system, which endows the system with maintainability and manageability characteristics, based on the current state of hospital management and national medical and health management standards.

## Figures and Tables

**Figure 1:** The composition of the nursing information system.

**Figure 2:** Topology diagram of medical monitoring data recognition algorithm scheme.

**Figure 3:** Sample loss.

**Figure 4:** The impact of different integration scales on the accuracy of the classifier.

**Figure 5:** Comparison of statistical error rates of different models.

**Figure 6:** Comparison of statistical time of different models.

**Figure 7:** Different initialization sequence.

**Figure 8:** The relationship between the actual value and the calculated value of stepwise linear regression.

## Data Availability

The data used to support the findings of this study are included within the article.
